The article "An Exploration: Alzheimer's Disease Classification Based on Convolutional Neural Network" was retracted in 2023. Reasons: signs of a paper mill; compromised peer review; unreliable results or conclusions.

# An Exploration: Alzheimer's Disease Classification Based on Convolutional Neural Network

**DOI:** 10.1155/2022/8739960

**Published:** 2022-01-22

**Authors:** Monika Sethi, Sachin Ahuja, Shalli Rani, Deepika Koundal, Atef Zaguia, Wegayehu Enbeyle

**Affiliations:** ^1^Chitkara University Institute of Engineering and Technology, Chitkara University, Punjab, India; ^2^Department of Systemics, School of Computer Science, University of Petroleum and Energy Studies, Dehradun, India; ^3^Department of Computer Science, College of Computers and Information Technology, Taif University, P.O. BOX 11099, Taif 21944, Saudi Arabia; ^4^Department of Statistics, Mizan-Tepi University, Ethiopia

## Abstract

Alzheimer's disease (AD) is the most generally known neurodegenerative disorder, leading to a steady deterioration in cognitive ability. Deep learning models have shown outstanding performance in the diagnosis of AD, and these models do not need any handcrafted feature extraction over conventional machine learning algorithms. Since the 2012 AlexNet accomplishment, the convolutional neural network (CNN) has been progressively utilized by the medical community to assist practitioners to early diagnose AD. This paper explores the current cutting edge applications of CNN on single and multimodality (combination of two or more modalities) neuroimaging data for the classification of AD. An exhaustive systematic search is conducted on four notable databases: Google Scholar, IEEE Xplore, ACM Digital Library, and PubMed in June 2021. The objective of this study is to examine the effectiveness of classification approaches on AD to analyze different kinds of datasets, neuroimaging modalities, preprocessing techniques, and data handling methods. However, CNN has achieved great success in the classification of AD; still, there are a lot of challenges particularly due to scarcity of medical imaging data and its possible scope in this field.

## 1. Introduction

AD is the degenerative disease that is most commonly known and progresses steadily. The age-by-age prevalence rate has been growing over the years, and interest in dementia-related research has grown worldwide. AD is one of the most well-known diseases among the old populace, and it confers adverse symptoms of dementia, including problems of memory (like intuition, recollecting, arranging, and judgment) [1]. The reported incidence rate is around 2 percent of the total at 65 years of age and 35 percent of the total or above at the age of 85. If lifespan increases, the percentage of people with AD increases dramatically. In 2006, there were around 26.6 million AD people reported. It is predicted that by 2050, this number would reach 0.1 billion [2]. It leads the hippocampus and cerebral cortex to reduce and the cerebral ventricles to enlarge. The intensity of all these disruptions depends on the stage of the disease. The significant shrinkage of the hippocampus and cerebral cortex and the enlargement of the ventricles could be seen in brain scans (MRI images) during the latter AD cycle [3, 4]. Early patients with AD are referred to as having Mild Cognitive Impairment (MCI), but not all MCI patients may be subject to AD. MCI is an intermediate stage from healthy to AD, wherein an individual has gentle changes in a psychological capacity that are evident to the individual influenced and to family members only. Progression time ranges around six months to three years, and yet, a year and a half is popular. MCI patients are categorized as either MCI Converters (MCIcs) or MCIs (MCIs), which indicate that they would have converted to AD for a year and a half or not. Besides that, there are similar subgroups of MCI that are less addressed in previous studies, and those subgroups are early MCI (i.e., eMCI) and late (i.e., lMCI) [5].

AD detection depends on a clinical assessment just like an extended meeting of the patient and their family members [6, 7]. In any case, “a ground truth” conclusion of AD must be rendered through a post-mortem examination, which is scientifically not helpful. Patients need some other basis to declare AD without ground truth information. Such criteria could improve our comprehension of AD and make finding feasible for living patients [8]. There is no commonly acknowledged remedy for AD, but there are a few remedies for postponing its course. It is also important to recognize early MCI subjects who are at risk of conversion to AD. The finding of AD depends basically on various factors, for example, hereditary data and demographics, neuropsychological tests, cerebrospinal fluid (CSF) biomarkers, and brain scans. In particular, the neuroimaging innovations, such as structural and functional magnetic resonance imaging (sMRI and fMRI), diffusion tensor imaging (DTI), single-photon emission tomography (SPECT), and positron emission tomography (PET), have been generally and effectively implemented in the investigation of MCI and AD. In sMRI, the radio frequency waves and magnetic fields are utilized [4] to take organ, bone, and tissue 3D images of the human body. In fMRI, changes related to blood flow are reflected. PET is a functional imaging technique that makes the use of radiopharmaceuticals that are injected into the bloodstream or inhaled directly. SPECT is a nuclear imaging test that combines both the Computed Tomography (CT) and radioactive tracers. SPECT examination is more affordable than PET. DTI is the advanced MRI method that gives detailed information on tissue microstructure. The choice of the neuroimaging methodology largely relies upon the seriousness of the diseased condition; for instance, where MRI could not uncover any cerebrum modifications, other modalities like PET, SPECT, or fMRI can examine the metabolic irregularities and DTI could be utilized for exploring the microstructural disturbance of the white matter (WM) [9].

Two of the most widely encountered indicators for the detection of AD are the Clinical Dementia Classification (CDR) and the Mini-Mental State Examination (MMSE) even though it ought to be noticed that utilizing these criteria as ground truth marking for an AD might be inaccurate. In light of the criteria referenced over, the detailed correctness of the clinical conclusion of AD contrasted with posthumous findings is in the scope of 70–90%. Regardless of its constraints, a clinical determination is the best accessible reference standard [5]. There is a requirement for a classification model unbiased by the radiologist, which should be able to differentiate AD. As of now for AD, no cure is available. So, it is of immense interest to create treatments to postpone its growth [10], particularly if AD can be analyzed at a beginning time where those treatments would have the most effect. In this manner, the exact and early classification of AD or MCI has a vital role in future treatment and patient care. However, it is as yet a difficult issue for precise and early diagnosing of AD/MCI.

Many computer-aided systems have been developed by researchers for accurate disease diagnosis. From the 1970s to the 1990s, they have created a rule-based expert framework, and from the 1990s onwards, supervised models [11] have been developed by them. To train supervised models, the features are extracted from the task-specific images [12]. Extracting these features requires human specialists that usually need a lot of effort, time, and funds. So, it is the biggest challenge for the data scientists to deal with. However, with the development of deep learning models, it is feasible to extract features directly from imaging data without human intervention. Thus, researchers are putting their attention on developing the deep learning model to diagnose the disease accurately. For various medical image analysis problems such as CT scans, MRIs, X-rays, ultrasounds, and sentiment analysis [13], deep learning models have attained significant success [14]. It has demonstrated notable results for distinct disease detection and classification in the domain of the lungs, abdomen, brain, cardiovascular, retina, and so forth.

As the most generally used design of DL, CNN has attained a lot of focus on account of its triumph in the area of image analysis and classification [15, 16]. But still, it is a big challenge for the researchers to diagnose AD using DL [5] due to less acquisition and errors in preprocessed medical images, inadequate knowledge especially in recognizing the Regions of Interest (ROI) within the cerebrum, imbalanced class subjects in the dataset, inaccessibility of dataset, and the low difference between different classes in various phases of AD. At times, the signs that separate AD, e.g., hippocampus shrinkage, can be noticed in a typical normal brain in old age, and as compared to natural images, the medical images are complex.

This paper is aimed at studying the cutting edge applications of CNN for the AD diagnostic on both single and multimodality brain scan data, and above all, what is the procedure to classify AD from the first to the last step? We have attempted to study a comprehensive research in this area to understand all the work that CNN has performed on single or multimodality neuroimages. Our purpose was also to evaluate how efficiently the CNN model could identify AD and its built-in capabilities to extract features that could boost the overall model's performance.

The rest of the paper is structured as follows.  Section 2 outlines briefly the CNN's architecture.  Section 3 introduces a procedure that is to be adopted to classify AD using deep learning particularly CNN followed by the subsections elaborating detailed information about each step. Finally, Section 4 depicts the limitations followed by the conclusion.

## 2. Architecture of CNN

CNN is a notable DL architecture or Feed Forward Network [17] that is modeled to perform a series of actions on multidimensional data like videos and images to achieve reasonable performance in different areas. Its architecture is motivated by the concept of the natural visual cortex suggested by Hubel and Wiesel [18] in 1959. It is built on the notion of receptive fields that is the area of an input image for which it looks for specific features similar to the animal visual cortex. In 1980, after the inspiration of Hubel and Wiesel's work, Fukushima [19] proposed Necognition which could be regarded as the CNN architecture's origin. In 1990, LeCun et al. set up the structure of CNNs by building up a multilayered artificial neural system which was termed LeNet-5, which was utilized to classify handwritten digits. Likewise other NNs, it could be trained with a back propagation algorithm which made it feasible to extract various patterns directly from raw images while eradicating the preprocessing steps required for feature extraction. However, at that time, it could not perform well on complex issues, for example, image or video classification, due to a shortage of training data and less computing resources.

Since the development of General Purpose GPUs and their utilization in AI [17], the field of CNN has experienced a revival stage. GPUs accelerated the computing techniques and made it feasible to train deep CNNs. In particular, in image recognition, Krizhevsky et al. presented a deeper CNN known as AlexNet which exhibited improvement in performance. AlexNet is fundamentally the same [20] as the LeNet-5 though more deeply in structure. With the achievement of AlexNet, numerous publications have been proposed to improve their performance. In particular, four publications are VGGNet [21], ResNet [22], GoogLeNet [23], and ZFNet [24].

CNN is a multilayered perceptron (MLP) composed of an input layer, many hidden layers, and lastly an output layer. The hidden layers further consist of many different other layers, namely, convolutional (C-layers), subsampling (S-layers), and fully connected (FC-Layers) [25].

C-layers are the fundamental aspect of the CNN model that is used to extract the low level to complex level features of the images. The learnable filters/kernels having a less receptive field are convolved with an input image through its full depth, evaluating the dot product between the input and filter, resulting in 2D feature maps corresponding to each filter. As an outcome, the network trains filters that activate only when it sees some specific features at some particular location in the input. S-layer lessens the data in each feature map that is obtained after the C-Layer while maintaining the most important features. There are typically a few rounds of C-layer and S-layer.

At last, an FC layer is utilized to take the outcomes from the C- and S-layers and convert them into a single long vector and use it to classify the various images into corresponding labels. The layered architecture of a standard CNN model is shown in Figure 1.

## 3. Method to Diagnose AD Using Neuroimaging Modality

AD is the most widely recognized degenerative disease, which grows gradually and causes brain cells to die. It is one of the common causes of dementia leading to a continuous decline in behavioral, social, and thinking abilities that disrupts the sufferer to function independently. Deep learning models have shown outstanding performance and do not need any handcrafted feature extraction over conventional machine learning algorithms. This paper expects to study AD detection using deep learning. Specifically, we investigated AD detection utilizing CNN to ascertain recent findings and emerging trends.

A schematic diagram of a computer-assisted AD diagnostic system using neuroimaging data is shown in Figure 2.

## 4. SLR Process

We first built up the study protocol at the initial phase of this SLR. The study protocol basically consists of phases such as setting up research questions (RQs), designing search query, study selection, data extraction and then lastly synthesis as illustrated in Figure 3.

In the first phase, we identified the set of research questions (RQs) based on the objectives for SLR. Then, in the second phase of SLR, focusing on the research questions, we devised a search query in such a manner that will help to answer our RQs and run that query on the different available databases like Google Scholar, PubMed, ACM Digital Library, and IEEE Xplore. In the primary phase study selection, we rejected many papers based on the title, abstract, and irrelevance and then downloaded only the number of papers that were nearly relevant to the study in step 4. In the 5th step, papers were studied in depth, and those papers that were not answering the research questions that were specified in step 1 were filtered out. In the data extraction phase, the useful information was extracted from each paper. Lastly, the extracted information was synthesized.

### 4.1. Research Questions

*RQ1*: what sorts of datasets are being used by authors to diagnose AD, and do they impact the accuracy of AD prediction?

*RQ2*: what kind of neuroimaging modalities are being used by the different research groups in AD classification? Do multimodalities over a single modality impact the performance of the classification?

*RQ3*: what sort of preprocessing techniques are available for neuroimaging data?

*RQ4*: what common data handling methods are being adopted by colleagues while feeding the data to the network, and how do these methods impact the performance of the network?

*RQ5*: what kind of CNN architectures (2D or 3D) are being implemented by researchers while classifying AD?

*RQ6*: does data augmentation and transfer learning methodology impact the accuracy of the network while the classification of AD?

### 4.2. Design Search Query Strategy

To answer the above-mentioned research questions, we efficiently explored publications where deep learning, specifically CNN, was utilized for the early diagnosis or classification of AD on different neuroimaging modalities. Specifically, we built an advanced query using keywords and joining them with OR and AND logical operators as follows: (“convolutional neural networks” OR “convolutional neural network”) AND neuroimaging AND (“Alzheimer's disease” OR Alzheimer's OR Alzheimer) AND (prediction OR classification). The query was then entered into four notable databases: Google Scholar, ACM Digital Library, PubMed, and IEEE Xplore between January 2012 and January 2020. Initially, a total of 2065 papers appeared in all of these databases (Google Scholar: 1890, PubMed: 78, IEEE Xplore: 45, ACM Digital Library: 52).

### 4.3. Selection Criteria

At first, the duplicate papers that were appearing on more than one resource were removed. After removal of duplicates, a total of 2065 research papers were filtered, and relevant papers were considered. The details are shown in Table 1. The studies were shortlisted on the basis of title, abstract, and conclusion. The results were studied, and then, inclusion and exclusion criteria were applied to these studies. The papers based on AD using CNN were included for the study. The papers not in English were also excluded from the survey. After performing inclusion and exclusion criteria, finally, 48 studies have been considered for the study.

*Step 1*: search through four notable databases separately and then gather the returned papers after excluding the duplicates.

*Step 2*: scan the reference lists of the relevant papers to find extra relevant papers and then, if any, add them into the set.

Searching and downloading studies is divided into two parts. Primarily, there are two options: Our primary search process consisted of the following phases. The first step is to identify key phrases from research questions. Analyze the terms used in step 1 and their synonyms. Boolean OR may be used to find synonyms and alternate spellings, while Boolean AND can be used to combine significant search words. With respect to the secondary search phase, we examine the references to identify main studies that were missed or neglected during the primary search phase and choose them for further selection.

SLR needs a thorough search of every single applicable source. Hence, we defined the search task and divided it into two. The complete search and selection process is shown in Figure 4.

### 4.4. Data Extraction

Extracted data from all the considered studies are summarized below in Table 2. In particular, we extracted the data required to answer the research questions mentioned above. Not every selected study provides answers to all the five research questions. For ease of tracing the extracted data, we explicitly labeled each study with the IDs of the research questions to which the study can provide the corresponding answers.

### 4.5. Synthesis

The set of research questions covered by the relevant papers identified in this study is shown in Table 3.

#### 4.5.1. Current Trends of Dataset in Prediction of AD

Various public datasets are available to assist the researchers to conduct their research in the area of AD classification. Public datasets, such as ADNI, MIRIAD [68–70], AIBL, and OASIS, are the commonly used datasets in this area of research. These datasets generally include the various types of neuroimaging modalities such as MRI, fMRI, PET, SPECT, cognitive and clinical assessments, and demographic information of the patients. The studies are aimed at testing the feasibility of using various brain scans as an outcome measure for clinical trials of AD treatments.

Among all mentioned datasets, ADNI is being vastly used standalone or with the combination of non-ADNI by few researchers [43] as shown in Figure 5. In 2003, pharmaceutical private companies, NIA, FDA, and NIBB, launched ADNI. The North American-based examination is expected to recruit 800 adults in total (around 200 adults with NC and early AD each and around 400 individuals with MCI). These individuals are followed by companies for two to three years. All subjects of ADNI are recruited from more than 50 sites across Canada and the US. The first purpose of ADNI is to check whether neurological and clinical assessments, genetic, PET, and MRI neuroimaging modalities can be joined together to measure progressive stages of AD.

OASIS is a project to provide free datasets to the scientific community that includes both longitudinal and cross-sectional MRI data of 150 and 416 subjects, respectively. The longitudinal datasets include both demented and nondemented elderly people's data within the age of 60 to 96. Whereas, the cross-sectional datasets include MRI data of demented and nondemented individual's data of young and aged people with their age lying between 18 and 96. For training and testing goals, a finite number of studies utilized separate datasets. In [71], the authors used OASIS MRI data for training the CNN model, and separate MIRIAD MRI data were utilized in the testing phase. Very few researchers have also used their private datasets with public datasets [29].

#### 4.5.2. Usage Comparison Based on Modality

Over the past decade, neuroimaging techniques have played an important role in the investigation of AD. At first, CT scan and after that MRIs were utilized to preclude different reasons for dementia. But nowadays, a variety of neuroimaging modalities including structural as well as functional MRI, FDG-PET, and DTI have exhibited changes of features in the brain images of AD sufferers.

MRI is one of the most famous strategies; noninvasive clinical imaging methodology is utilized to capture the inward body structures [10]. It utilizes radio frequency and magnetic fields to create virtually the complete images of tissues, bones, and internal structure of the brain. Basic MRIs are regularly used to identify the local atrophy of the brain and comprehend cerebrum anatomical changes. Consequently, for AD diagnosis, they are considered as an efficient biomarker. Changes identified with the bloodstream are reflected in fMRI [4]. PET is a functional imaging method that utilizes radiotracers that are inhaled directly or injected into the bloodstream.

Many of the studies had done work on single modality only either on PET, MRI, DTI, or fMRI to classify AD. And only a few of the researchers worked on multimodalities with the consideration that fusion of modalities provides complementary information and enhances the performance for AD classification. But only a few studies [40, 44, 60] have made a comparison of using single modality vs. fusion modalities in their research work. In [40], the authors achieved high accuracy for AD vs. HC classification with a fusion of two modalities, MRI and PET, as compared to working only with a single modality, either MRI or PET images. In the same way in [44], when MRI and PET images were considered together, the accuracy reached the level of 91% for AD/HC classification that is almost 9% and 1% higher than when only single modality MRI or PET images were considered separately. In [60], 92% accuracy was achieved for discriminating AD from HC when two modalities MRI and PET were used together. In their experiment, the authors even considered the same number of subjects as 585 for both modalities while in fusion. The prevalence of using neuroimaging modalities for AD classification is shown in Figures 6 and 7.

#### 4.5.3. Preprocessing Techniques for Neuroimaging Data

After acquiring the neuroimaging modalities, there is a need to know how these modalities are utilized in DL architectures by various groups of researchers for the diagnosis of AD. Before analysis, the neuroimaging modalities undergo a series of preprocessing steps that are required to improve and prepare the data for further usage. And this is one of the mandatory steps, as the complete triumph of an automatic diagnostic system relies emphatically upon how effectively the preprocessing steps are considered. Nowadays, there are numerous tools available that are used for neuroimaging data preprocessing, for instance, FSL, FreeSurfer [15], DARTEL [43], and SPM [29, 31, 43].

With the applications of DL strategies, images require less or no image preprocessing [43]. However, many researchers still employ preprocessing techniques on different modalities before the actual analysis to be conducted. These techniques are skull stripping, intensity normalization, tissue segmentation, registration, motion correction, and Gradwarp.

Skull stripping is the preprocessing technique opted by [15, 38, 42, 45, 49, 71, 72], used to remove the unnecessary details of nonbrain regions such as the skull, muscle, fat, and eyes of the brain images as these parts are not affected by the AD disease.

Different parameters or scanners would be utilized while taking neuroimages for the same or different subjects over time, which may further bring huge variations in intensities. This could greatly impact the performance of subsequent processing techniques and analysis as well. So, it requires intensity normalization, which is a process by which the range of voxel and pixel intensity values is changed to a referenced scale. The purpose is to achieve a consistent range of intensities for the similar structures of the images. Nonparametric nonuniform intensity normalization (N3) is a widely used method [15, 42, 45, 51] to correct MR images by eliminating intensity nonuniformity of the image. For AD classification, other researcher groups [51, 72] have used Gaussian filter with 8 mm and 5 mm FWHM, resp., for spatial smoothing.

Another method for preprocessing is the tissue segmentation utilized by [3, 43] that is aimed at dividing a brain image into different segments, for instance, white matter (WM), gray matter (GM), and cerebrospinal fluid (CSF) to compute their volumes. In AD, GM may lose volume before WM. As compared to the normal control, an increased GM atrophy rate of about 2 percent/year was seen in AD subjects [73]. It may improve the precision of the diagnosis and thus act as an early diagnostic biomarker, especially for AD [74]. Image registration technique is used by [72], which means to align two or more images with the other image designated as fixed or reference image using the Montreal Neurological Institute standard space (MNI152). In medical imaging, it enables us to join data from different neuroimaging modalities that are known as coregistration [51]. For instance, multiple modalities MRI, PET, CT scan, or SPECT are combined to have complete information about the subject. In [43], by using the SPM and DARTEL registration method, 3D T1-weighted images from both ADNI and MILAN datasets were normalized to the MNI space. The AC and PC are two important brain structures and crucial landmarks used in [45] for reorientation. Another widely used preprocessing technique is the motion correction utilized in [72] to suppress the motion artifacts.

#### 4.5.4. Performance Comparison Using Different Types of Data Handling Methods

To classify the subjects into different categories (like HC, AD, or MCI), the features are extracted from the preprocessed neuroimages. The classification process includes multiple steps including feature extraction, selection, and reducing the number of features (i.e., dimensionality reduction), and finally, based on the reduced selected features, classification is performed. With the advent of neural networks, primarily CNN, it has become possible to integrate all these steps into a single system and be able to automatically and adaptively learn the hierarchy of features from low to complex levels by back propagation [74]. Still, for the active researcher, it is the biggest challenge to manage the whole neuroimaging modality. By utilizing the different ways [75] such as slice, ROI, patch, and voxel-based, the neuroimages are handled by the researchers as shown in Figure 8.

*(1) Slice Based*. To diagnose AD, axial view planes of the brain scans are widely used by active researchers. The first ten slices of MRI along the axial plane were discarded [72] by Saman Saraf, as no useful information for classification was found in those slices, and the rest were stacked together. The same author discarded the last 10 slices along the axial plane and where the sum of pixel the intensity value approaches zero. The authors of [35], to diagnose each group from the GM part of scans, removed both the start and end slices.

In [76], also the middle axial slices were considered for ADNI 660 MRI scans. Luo et al. [28] just extracted the middle patches numbered from 25 to 31 for every MRI along with 5 adjacent slices. Rather than random slice extraction, an image entropy approach was used by authors in [15, 59], to extract the most informative slices from the 3D neuroscans.

To diagnose AD, coronal view planes of MRI neuroscans were considered by the authors in [2, 50] as it covers the main 3 regions of the cortex, ventricles, and hippocampus.

Researchers in [56] showed the influence of random selection and precise selection of slices along the 3 planes, and the best accuracy was obtained with the coronal slices at 95%.

To train the network, only 5 middle sagittal slices from the hippocampus region were considered by the authors in [26]. To diagnose AD, the authors in [11, 30, 71, 77, 78] considered all three views of 3D neuroimages with the assumption that they may contain complementary information.

*(2) Patch Based*. As there is no 3D spatial information in the slice-based approach, few studies focused on the patch-based technique. A patch is a 3D cube that does not require any ROI identification. The entire brain area is split into compact-size patches in this procedure, and from these patches, the features are derived. Since learning is from the entire brain region, pathologies linked to disease are best captured, leading to better diagnostic results. But still, selecting the most insightful patches for creating image-level (global) and patch-level (local) discriminatory features is a huge challenge. Several researchers have used this approach for AD discrimination [31]. In two different studies [42, 51], the authors have used 27 large 3D patches of size (50∗41∗40) from the entire brain images of size (100∗81∗80). In another study [40], patches of size 5∗5∗5 from MRI and PET neuroimages were extracted. In their next study [39], the authors experimented with three different sized patches as *v* = 3, 5, and 7.

*(3) ROI Based*. The brain is composed of many organs that are intended to execute separate functions, and AD is not correlated with all those organs. Consequently, the ROI strategy mainly focuses on the subpart of the brain that is impacted during AD rather than working with the whole brain image to diagnose AD [45]. Furthermore, this strategy needs domain knowledge of medical research in the area of identification of ROI that are influenced by AD.

In [45], the researchers proposed, with their experimental findings, the top 10 brain regions that have a major influence on the diagnosis of AD. On the other hand, the authors in [71] extracted slices from specific regions influenced by AD. The researchers in [26, 45] extracted only one hippocampal as an ROI, and volume of the cortex, ventricles, and the hippocampus as 3 different ROIs were considered in [2]. In a similar way in [79], to diagnose various stages of AD, the peers extracted only GM as a ROI from the MRI scan. Hippocampi as an ROI from multimodality neuroimages (DTI and sMRI) were considered by the researcher group in [78]. In [80], from each of the 3D PET images using the 2nd edition of the AAL-2 atlas with 120 ROIs, the authors derived ROI-mean PET signals.

*(4) Voxel Based*. Voxel-based approaches, opposed to the ROI methodology, are unbiased of any assumption and are simple to employ for brain structure research. The classification is done regardless of the slice or patch level where the entire MRI is used at once and spatial information is preserved. The number of samples per subject is usually very small from very few hundreds to thousands in the 3D voxel-based process, however, compared to the number of features to optimize that lead to over fitting problems [11]. To address the issue of high dimensionality as used by Ortiz and colleagues [80], the preselection approach for the voxel may be implemented independently on each modality. As illustrated in the table, very few studies have used this method.

#### 4.5.5. Performance Comparison 2D CNN/3D CNN

For AD classification, many studies have utilized 2D CNN with an input of 2D slices extricated from 3D MRI images. In this section, few studies are examined for those who have used 2D CNN with their architecture, adopted architecture, or transfer learning. For each of the studies, which of the modality coworkers have opted and the type of the input to the network are mentioned.

Gunawardena and colleagues [2] used several 2D CNNs consisting of two C-layers, one S-layer, and an FC layer for each of their experiments on 2D coronal view slices of the MRI images. 2D CNN architecture consisting of 2 C-layers on 2D sagittal planes [26], in the center of the hippocampal area of MRI data, was also used by Aderghal et al. The authors extended their architecture in [27], and all the three views, axial, coronal, and sagittal, from the same subject's brain were fused and the classification outcome using a majority voting technique was obtained. Luo and colleagues [28] used 7 2D CNNs for 7 sections numbered from 25 to 31 consisting of five neighborhood slices of 3D MRI brain images for AD recognition. Wang et al. also used 8-layered 2D CNN on the sagittal view of MRI data for AD recognition [29]. Three different pooling functions (average, max, and stochastic) and activation functions (ReLu, leaky ReLu, and Sigmoid) were experimented. The leaky ReLu activation function and max-pooling gave the best results for image classification.

In numerous studies, 2D CNN architecture based on AlexNet, LeNet, GoogleNet, and ResNet was adjusted and widely used. For example, Sarraf and colleagues chose 2D CNN based on LeNet-5 architecture and adjusted it for fMRI data [33, 72] and MRI (GM 2D slices) [34]. The authors adopted LeNet and GoogleNet for both fMRI and GM 2D slices of MRI data for AD diagnosis [3]. As compared to the LeNet model, the GoogleNet model showed better accuracy.

In 2D CNNs, to evaluate features from the spatial dimensions, convolutions are applied on the 2D feature maps only. There is a spatial relationship in the image since MRI neuroimages are 3D in nature. To gain those spatial correlations of 3D, 3D CNNs have been employed in numerous studies, and according to the researchers, 3D CNNs give better performance than 2D CNN during imaging classification. For example, in [44], the authors designed 3D CNN to combine the features from a hippocampal area of both the modalities T1-weighted MR and FDG-PET to classify AD. In [32], Payan and coworkers employed both 2D CNN and 3D CNN with pretrained SAE on the same dataset and obtained better accuracy in the case of 3D CNN as compared to the 2D CNN. Their experiments showed that a 3D method had the potential to grasp the 3D local patterns leading to high classification performance. Li et al. proposed the integration of two multimodel convolutional networks, namely, CNN and CAE (3D), on MRI images for AD classification [38]. Two 3D CNNs were pretrained using SAE on MRI and PET modalities separately and then combined using an upper fully connected layer to make classification on AD [39]. A comparison in terms of performance was done between two 3D CNN models with or without SAE (for pretraining) [40]. It has been concluded that the 3D CNN model achieved better accuracy with SAE. In [41], Khvostikov and coworkers employed 3D CNN for both left and right hippocampal ROI of both modalities sMRI and DTI followed by fully connected layers to combine them for classification. In another paper [42], a set of 3D CNNs were employed to extract the features from each of the local patches of the MRI modality. In [43], Basaia and colleagues designed straight 3D CNN architecture for AD classification.

In numerous studies, 3D CNN architecture based on already existing networks such as AlexNet, LeNet, GoogleNet, and ResNet has been adjusted and widely used. Korolev et al. employed 3D CNN architecture [46] based on ResNet and VGGNet for the task of classification of brain MRI images. In [47], Karasawa et al. employed 3D CNN using a cubic filter based on ResNet architecture on 3D MRI brain scans. Cheng et al. designed a fusion of 2 CNN models (2D CNN and 3D CNN) named as cascaded CNN in two of their studies [10, 48].

#### 4.5.6. Impact of Data Augmentation and Transfer Learning Approaches

An AD sufferer's neuroimaging datasets are generally of little size as compared to any other datasets. Because of the enormous number of learned parameters from a small dataset, DL models tend to overfit. To overcome this issue [14], data augmentation (DA) is the technique used to generate images from the existing training dataset samples, thus increasing the size of data to be used for training and testing. It can be classified as a transformation or data synthesis technique.

Data augmentation techniques have been used by many studies to improve the classification performance [11, 29, 58, 76]. In [76], binary classification for AD/CN the accuracy with data augmentation was increased by about 2.5% and 0.7% for ternary classification AD/MCI/CN.

Despite the fact that CNNs have performed extraordinarily well in medical image analysis for classification in the last couple of years, the training of these architectures on a ground-level basis has few issues [15], like these architectures need a colossal amount of labeled data for training especially for medical imaging areas where it is too costly and sometimes hard to procure adequate data. It also requires a huge amount of computational resources such as GPUs and hyperparameter optimal tuning which may otherwise create underfitting or overfitting issues leading to the poor performance of the model. To handle these issues, analysts came up with an effective methodology called transfer learning [81]. Transfer learning is an ML technique where an already developed model for a particular task is reutilized as a baseline for other tasks. There are three strategies for the transfer learning method, namely, train the full model from scratch (requires a huge amount of dataset for training), train some layers and freeze others, and freeze the convolutional base (responsible for feature engineering). In [50], instead of using a Gaussian or random initialization, the weights of the 16-layered VGGNet were used to initialize the 2D CNN's filters. Similarly, a statistical model P_F_S_E_CT_L_ built on the transfer learning approach is implemented on sMRI brain slices for ternary classification (AD vs. CN vs. MCI) in [15]. They utilized pretrained VGG-16 for transfer learning and feature extraction. Although VGGNet-16 was trained on natural images, it was still capable of extracting useful features for their task of classification. However, the dataset employed for pretraining often affects the impact of transfer learning on the performance of the network. In [58], CNN's integration with a pretrained model using the OASIS dataset outperformed CNN's integration with a pretrained model using the LIDC dataset for AD classification. In [14], for learning features from a small OASIS dataset, Islam and Zhang utilized a pretrained Inception-V4 model to set the hyperparameters of their network rather than random initialization. To fit the input MRI data to the Inception-V4 model, they transformed the input size to 299∗299∗1. In their other research [12], three DenseNet networks varying with depths as 121-161-169 pretrained using the ImageNet dataset were utilized and later fine-tuned for MRI images of the OASIS dataset. In [56], coworkers applied three modified DenseNet architectures (121-169-201) to the pretrained 2D CNN model on image slices as the input, and DenseNet-121 outperformed DenseNet-169 and DenseNet-201. In [59], the authors used a very small-sized training dataset with a pretrained Inception-V4 model on slice-based MRI data and achieved comparable accuracy with [3]. Both VGG-16 models from scratch and with transfer learning were used for comparison. It has been observed that when it was trained using transfer learning, it resulted in significant improvement in accuracy for classification than from scratch. The reason for poor performance in VGG-16 from scratch was it used a small-sized training dataset [59].

## 5. Discussion and Limitation

A direct comparison among outcomes of the different studies is impacted by several parameters such as different datasets as well as different cohort sizes and different neuroimaging modalities; some researchers considered only one modality (MRI), and few of the researchers opted for multimodalities for their research work and different preprocessing techniques as well as different data handling methods. The most commonly used dataset and modalities for AD classification are ADNI and MRI neuroimages, respectively. However, managing the entire neuroimaging modality has been the most difficult issue for the active researcher. The neuroimages are processed by the researchers using several methods such as slice, ROI, patch, and voxel based. It has been noted that ROI- and patch-based data handling approaches are much more effective compared to slice- and voxel-based processes. In comparison to the 2D CNN, 3D CNN is being employed to gain spatial correlations of 3D MRI images, and they provide better performance. Regardless of the fact that CNNs have performed remarkably well in medical image analysis for classification over the last few years, the learning of these frameworks on a ground-level basis has a few challenges, such as these designs require a massive amount of labelled data for training, especially in medical image processing areas where it is too highly priced or sometimes hard to obtain sufficient information. It also demands a massive proportion of computational services including GPUs, hyperparameters, and effective tuning that may also possibly result in underfitting or overfitting issues, leading to a poor prediction model. To address these challenges, analysts devised an efficient process known as transfer learning. So, transfer learning is being utilized to improve the performance of the network as well as to overcome the issue for the requirement of huge amount of data to train deep learning models.

There is no standard way to select the dataset, and it may affect the performance of the classifier. Moreover, researchers have used different CNN models with variations of a different set of C-layers and FC layers. They have not provided any clear way of how they have selected and designed their models to classify AD. Another main limitation and challenge is the use of multimodality as it is very hard to join the features from different modalities as some modalities are not complete for each subject and there is missing data. In the case of the data handling methods, recognizing the specific ROI and patch that contains the main features for the AD is very hard to get and it requires expert knowledge.

## 6. Conclusion

AD is most widely recognized as an irreversible degenerative disorder, which grows slowly and leads to neuronal cell death. In comparison to the conventional machine learning approach, recently, the deep learning approach specifically CNN has gained huge success in the field of a medical domain in the classification of AD, and it does not need any handcrafted feature extraction technique. In this paper, we discussed the method adopted for AD classification while using CNN and what kinds of datasets were available publically, what type of neuroimaging data modalities were available, what sort of preprocessing methods were used, and what sort of data is inputted into the CNN. The advantages of using multimodalities over single modality and the role of data augmentation and transfer learning were discussed for classification accuracy of the CNN model. Comparison among the accuracy results of chosen studies are influenced by numerous factors, like all had utilized a different set of subjects, neuroimaging modalities, modality preprocessing procedures, and different data handling methods. So, it is just impossible to conclude which approach is the best one. However, we found some common points: the widely used modality to classify AD is MRI and multiple modalities over a single modality give better accuracy results for AD classification with the consideration that these provide complementary information. Patch and ROI data handling methods are much more efficient as compared to slice- and voxel-based techniques. 3D CNN is being employed to gain spatial correlations of 3D MRI images, and they provide better performance in comparison to the 2D CNN. Other key factors to enhance the performance of the network are to use data augmentation and transfer learning.

## Figures and Tables

**Figure 1:** Layered architecture of CNN.

**Figure 2:** A schematic diagram using computer-assisted AD detection procedure.

**Figure 3:** Method adopted for SLR.

**Figure 4:** Search and selection process.

**Figure 5:** Prevalence of using dataset.

**Figure 6:** Prevalence of multimodality vs. single modality.

**Figure 7:** Neuroimaging modality prevalence.

**Figure 8:** Prevalence of data handling techniques.

**Table 1:** Published papers to detect AD since 2012 using CNN.

Year	Papers that appear	Rejected based on the title	Downloaded	Rejected based on abstract, thesis, book chapter	Included in survey
2012	12	12	0	0	0
2013	13	12	1	0	1
2014	16	15	1	0	1
2015	46	43	3	2	1
2016	114	106	8	4	4
2017	308	286	22	5	17
2018	653	606	47	35	12
2019	851	819	32	27	5
2020	35	33	2	1	1
2021	17	6	11	5	6
Total	2065	1938	127	79	48

**Table 2:** Characteristics of each of the study included in survey.

Ref no. (year)	Model	Data handling approach	Preprocessing techniques	Modality		Dataset	Cohort or subjects					Classification				Data augmentation	Transfer learning
				1	>1		AD	MCI		NC	Total	Binary			Multiclass (3-way or 4-way)		
								cMCI	ncMCI			AD vs. HC	AD vs. MCI	MCI vs. HC			
[2] (2017)	SVM	Slice based	Noise removal, linear normalization, image enhancement	MRI	—	ADNI	—	—	—	—	—	Sensitivity: 95.3% specificity:71.4%				—	No
	2D CNN						7	14		15	36	Sensitivity: 96% specificity:98%				—	
	2D CNN						9	16		11	36	Sensitivity: 95% specificity:98%				—	
[26] (2017)	2D CNN	Slice based	Image alignment, image normalization	MRI	—	ADNI	188	399		288	875	82.20%	62.50%	66%	—	Yes	No
[27] (2017)	2D CNN	Slice based	Geometric normalization for registration	MRI	—	ADNI	188	399		288	875	91%	—	—	—	Yes	No
[28] (2017)	2D CNN	Slice based	Gradwarp, B1 nonuniformity, N3	MRI	—	ADNI	47	—		34	81	93%	—	—	—	Yes	No
[29] (2018)	2D CNN	Slice based	Skull stripping, spatial normalization and smoothing	MRI	—	OASIS+community advertisements	28+70	—		98+0	196	97.65%	—	—	—	Yes	No
[11] (2018)	2D CNN	Slice based	—	MRI	—	OASIS	—	—		—	416	—	—	—	93.18%	Yes	No
[30] (2018)	2D CNN+RNN	Slice based	No segmentation and rigid registration	FDG-PET	—	ADNI	98	146		100	339	—	—	78.9%	—	Yes	No
[31] 2013	Sparse encoder+2D CNN	Patch based	Normalization using statistical parametric mapping (SPM)	sMRI	—	ADNI	200	411		232	843	93.8%	86.3%	83.3%	78.2%	Yes	Yes
[32] (2015)	Sparse encoder+2D CNN	Slice based	Normalization using statistical parametric mapping (SPM)	MRI	—	ADNI	755	755		755	2265	95.39%	82.24%	90.13%	85.53%	Yes	No
	Sparse encoder+3D CNN	Voxel based										98.85%	86.84%	92.11%	89.47%		
[33] (2016)	2D CNN	Slice based	Motion correction, skull stripping, and spatial smoothing	rs-fMRI	—	ADNI	28	—		15	43	98.85%	—	—	—	Yes	No
[34] (2016)	2D CNN	Slice based	Skull striping, registration, spatial smoothing	MRI	—	ADNI	211	—		91	302	98.84%	—	—	—	Yes	No
[3] (2017)	2D CNN	Slice based	Skull stripping, spatial smoothing, registration using MNI	MRI	—	ADNI	211	—		91	302	98.84%	—	—	—	Yes	No
		Subject based										100%					
		Slice based		rs-fMRI			52			92	144	99.9%					
		Subject based										97.77%					
[35] (2017)	2D CNN based	Slice based	Skull stripping and the GM segmentation	MRI	—	ADNI	33	22	49	45	149	—	—	—	4-way based	Yes	No
	GoogleNet														98.9%		
	ResNet-18														98.01%		
	ResNet-152														98.14%		
[36] (2016)	3D CAE+3DCNN (3D ACNN)	Voxel based	No preprocessing	MRI	—	CADDementia MRI and validated on ADNI	70	70		70	210	97.60%	95%	90.80%	89.1% (3-way)	No	Yes
[37] (2016)	Deeply supervised adaptive 3D-CNN (DSA-3D CNN)	Voxel based	Used no preprocessing techniques	MRI	—	ADNI MRI and validated on CADDementia	70	70		70	210	99.30%	100.00%	94.20%	94.8% (3-way)	—	Yes
[38] (2017)	3D CNN+3D CAE	Voxel based	Skull stripping and cerebellum-removal (after an intensity inhomogeneity correction)	MRI		ADNI	199	—		229	428	88.31%	—	—	—	—	—
[39] (2017)	SAE+3DCNN	Patch based (patch size = 3)	Anterior commissure posterior commissure (AC-PC) correction, skull stripping, and cerebellum removal	—	MRI and PET	ADNI	145	192		172	509	93.14%	82.36%	89.47%	86.13%	Yes	Yes
		Patch size = 5										93.59%	82.92%	93.25	89.24%		
		Patch size = 7										91.06%	83.75%	91.14%	87.53%		
[40] (2017)	3D CNN	Patch based	Skull stripping, cerebellum removal, AC-PC correction	MRI	—	ADNI	145	—		172	317	80.62%	—	—	—	—	—
	SAE+3D CNN											85.24%					
	3D CNN			PET	—							81.93%					
	SAE+3D CNN											85.53%					
	3D CNN			—	MRI and PET							84.72					
	SAE+3D CNN											91.14%					
[41] (2018)	3D CNN	ROI based	Skull stripping, coregistration, spatially normalized	—	MRI+DTI	ADNI	48	108		58	214	85%	75%	66%	—	No	—
												96.70%	80%	65.80%		Yes	
[42] (2017)	3D CNN	Patch based	Correction of intensity inhomogeneity, skull stripping, and cerebellum removal	MRI	—	ADNI	199	—		299	498	87.15%	—	—	—	—	No
[43] (2019)	3D CNN	Slice based	Normalization using statistical parametric mapping and diffeomorphic anatomical registration exponentiated lie algebra (DARTEL)	sMRI		ADNI+non-ADNI (“Milan”)	294 + 124	253 + 27	510 + 23	352 + 55	1409 + 229	99.2% (with ADNI) 98.2% (with ADNI and Milan)	—	—	—	Yes	Yes
[44] (2019)	3D CNN	ROI based	—	MRI	—	ADNI	647	326	441	731	2145	81.19%	—	—	—	—	No
				FDG-PET	—							89.11%					
				—	MRI and FDG-PET							90.10%					
[45] (2019)	3D CNN	ROI based	AC_PC, tissue intensity inhomogeneity, skull stripping and cerebellum removal, registration	—	MRI and PET	ADNI	93	76	128	100	397	94.82%	—	4.5**—**	—	—	No
[46] (2017)	3D CNN based on VGGNet and ResNet	Voxel based	Skull stripping, spatially normalized	MRI	—	ADNI	50	43	77	61	231	88% (VGGNet)	—	—	—	—	No
[47] (2018)	3D CNN (based on ResNet)	Voxel based	—	MRI	—	ADNI	345	450		574	1370	94%	—	90%	87%	—	No
[48] (2018)	3D CNN followed by 2D CNN	Voxel based	No preprocessing	—	MRI and PET	ADNI	93	—		100	193	89.64%	—	—	—	Yes	No
[10] (2018)	3D CNN followed by 2D CNN	Patch based	No segmentation and rigid registration	—	MRI and PET	ADNI	93	76	128	100	397	93.29%	—	—	—	Yes	Yes
[49] (2014)	3D CNN	Patch based	Intensity inhomogeneity, skull stripping and cerebellum removal	—	MRI and PET	ADNI	198	167	236	229	830	92.875	—	76.21%	—	Yes	No
[50] (2017)	2D CNN	Slice based	Motion correction, skull stripping and, intensity normalization	MRI	—	ADNI	300	300		300	900	—	—	—	91.85%	Yes	Yes
[51] (2017)	3D CNN	Patch based	Intensity normalization and coregistration	PET	—	ADNI	93	—		100	193	92.20%	—	—	—	Yes	No
[52] (2018)	CaffeNet	Slice based	Gradwarp, intensity inhomogeneity correction, and N3 histogram peak sharpening	MRI	—	ADNI	—	157	150	457	764	—	—	—	87.78%	Yes	Yes
	GoogleNet														83.23%		
[53] (2018)	3D CNN	Voxel based	Registration, histogram matching	MRI+clinical assessment and genetic (APOe4)	—	ADNI	192			184	376	99%	—	—	—	—	No
[54] (2018)	2D CNN	Slice based	Spatially normalized, skull stripping	MRI	—	ADNI	150	129		112	391	95.91%	86.84%		89.76%	Yes	No
	3D CNN											96.81%	88.435		91.32%		
[55] (2018)	En3DCNN	ROI based	Nonuniformity (NU) intensity correction, motion correction, Talairach space conversion	MRI	—	ADNI	347	—		417	764	93.90%	—	—	—	Yes	No
[56] (2018)	2D CNN	Slice based	Skull stripping	MRI	—	ADNI	347	806		537	1690	94.97%	91.98%	74.7%	—	Yes	Yes
[57] (2018)	2D CNN	Slice based	Gradient unwarping, nonparametric nonuniformed bias correction	sMRI	—	ADNI	336	542		785	1663	95.45%	93.88%	95.39%	—	—	—
[15] (2019)	2D CNN	Slice based	Skull stripping, motion correction, and NU intensity normalization	MRI	—	ADNI	50	50		50	150	99.14%	99.3%	99.22%	95.73%	Yes	Yes
[58] (2017)	Expedited CNN	Voxel based	—	sMRI	—	ADNI	—	400		229	629	—	—	88.8%	—	Yes	With LIDC
														90.6%			With OASIS
[12] (2017)	2D CNN based DenseNet-121-161-169	Slice based	—	MRI	—	OASIS		—		—	416	—	—	—	93.18%	No	Yes
[59] (2017)	VGG-16 (from scratch)	Slice based	—	sMRI	—	OASIS	100	—		100	200	74.13%	—	—	—	Yes	Yes
	VGG-16 (transfer learning)											92.3%					
	Inception V4 (transfer learning)											96.25%					
[60] (2019)	3D CNN	Voxel based	Skull stripping, bias field correction, volumetric and affine registration	MRI	—	ADNI	—	—		—	585	73.76%	—	—	—	—	No
				PET	—						585	85.15%					
				—	MRI+PET						585+585	92.34%					
[61] (2020)	2D CNN	ROI based	Spatially segmented and normalized, skull stripping, coregistration	—	MRI+DTI	ADNI	115	106		185	406	93.50%	—	79.6%	—	—	No
[62] (2021)	3DCNN	Voxel based	Registration and segmentation	MRI	—	ADNI	146	146		256	548	—	89.3%	87.5%	—	No	No
[63] (2021)	DCNN, VGG-16, VGG-19	Slice based	Flipping, random zooming	MRI	—	OASIS	—	—		—	416	—	—	—	71%	Yes	Yes
[64] (2021)	Deep transfer ensemble (DTE)	Slice based	FWHM, segmentation, registration	MRI	—	ADNI	187	398		228	813	99%	98.7%	—	—	Yes	Yes
[65] (2021)	VGG DenseNet ResNet EfficientNet	Slice based	—	MRI	—	OASIS	—	—		—	416	—	—	—	72% 92% 93% 96%	Yes	Yes
[66] (2021)	AlexNet	Slice based	—	MRI	—	OASIS	—	—		—	664	—	—	—	96%	Yes	Yes
[67] (2021)	VGG-16	Slice based	3D to 2D conversion	fMRI	—	ADNI	18	—		36	54	99.9	—	—	—	Yes	Yes

**Table 3:** Research questions covered by the studies included this systematic study.

Study	Reference (year)	Research questions answered					
		RQ1	RQ2	RQ3	RQ4	RQ5	RQ6
1	[2] (2017)	Yes	Yes	Yes	Yes	No	Yes
2	[26] (2017)	Yes	Yes	Yes	Yes	Yes	Yes
3	[27] (2017)	Yes	Yes	Yes	Yes	Yes	Yes
4	[28] (2017)	Yes	Yes	Yes	Yes	Yes	Yes
5	[29] (2018)	Yes	Yes	Yes	Yes	Yes	Yes
6	[11] (2018)	Yes	Yes	Yes	Yes	Yes	No
7	[30] (2018)	Yes	Yes	Yes	Yes	No	No
8	[31] 2013	Yes	Yes	Yes	Yes	No	No
9	[32] (2015)	Yes	Yes	Yes	Yes	Yes	Yes
10	[33] (2016)	Yes	Yes	Yes	Yes	No	Yes
11	[34] (2016)	Yes	Yes	Yes	Yes	No	Yes
12	[3] (2017)	Yes	Yes	Yes	Yes	Yes	Yes
13	[35] (2017)	Yes	Yes	Yes	Yes	No	Yes
14	[36] (2016)	Yes	Yes	Yes	Yes	No	Yes
15	[37] (2016)	Yes	Yes	No	Yes	No	Yes
16	[38] (2017)	Yes	Yes	Yes	Yes	No	Yes
17	[39] (2017)	Yes	Yes	Yes	Yes	No	Yes
18	[40] (2017)	Yes	Yes	Yes	Yes	No	Yes
19	[41] (2018)	Yes	Yes	Yes	Yes	No	Yes
20	[42] (2017)	Yes	Yes	Yes	Yes	No	Yes
21	[43] (2019)	Yes	Yes	Yes	Yes	No	No
22	[44] (2019)	Yes	Yes	Yes	Yes	No	Yes
23	[45] (2019)	Yes	Yes	Yes	Yes	No	Yes
24	[46] (2017)	Yes	Yes	Yes	Yes	No	Yes
25	[47] (2018)	Yes	Yes	Yes	Yes	Yes	No
26	[48] (2018)	Yes	Yes	Yes	Yes	Yes	Yes
27	[10] (2018)	Yes	Yes	Yes	Yes	Yes	Yes
28	[49] (2014)	Yes	Yes	Yes	Yes	No	Yes
29	[50] (2017)	Yes	Yes	Yes	Yes	No	Yes
30	[51] (2017)	Yes	Yes	Yes	Yes	No	Yes
31	[52] (2018)	Yes	Yes	Yes	Yes	Yes	Yes
32	[53] (2018)	Yes	Yes	Yes	Yes	No	Yes
33	[54] (2018)	Yes	Yes	Yes	Yes	No	Yes
34	[55] (2018)	Yes	Yes	Yes	Yes	Yes	Yes
35	[56] (2018)	Yes	Yes	Yes	Yes	Yes	Yes
36	[57] (2018)	Yes	Yes	Yes	Yes	No	No
37	[15] (2019)	Yes	Yes	Yes	Yes	Yes	Yes
38	[58] (2017)	Yes	Yes	Yes	Yes	Yes	Yes
39	[12] (2017)	Yes	Yes	Yes	Yes	Yes	Yes
40	[59] (2017)	Yes	Yes	Yes	Yes	Yes	Yes
41	[60] (2019)	Yes	Yes	Yes	Yes	No	Yes
42	[61] (2020)	Yes	Yes	Yes	Yes	No	Yes
43	[62] (2021)	Yes	Yes	Yes	Yes	Yes	Yes
44	[63] (2021)	Yes	Yes	Yes	Yes	Yes	Yes
45	[64] (2021)	Yes	Yes	Yes	Yes	Yes	Yes
46	[65] (2021)	Yes	Yes	Yes	Yes	Yes	Yes
47	[66] (2021)	Yes	Yes	Yes	Yes	Yes	Yes
48	[67] (2021)	Yes	Yes	Yes	Yes	Yes	Yes

## Data Availability

There is no data used in this research.
